The article "The Association between Skull Bone Fractures and the Mortality Outcomes of Patients with Traumatic Brain Injury" was published in 2022. Journal: Emerg Med Int.

# The Association between Skull Bone Fractures and the Mortality Outcomes of Patients with Traumatic Brain Injury

**DOI:** 10.1155/2022/1296590

**Published:** 2022-06-07

**Authors:** Yu-Chin Tsai, Cheng-Shyuan Rau, Jin-Fu Huang, Yu-Min Chang, Kai-Jay Chia, Ting-Min Hsieh, Sheng-En Chou, Wei-Ti Su, Shiun-Yuan Hsu, Ching-Hua Hsieh

**Affiliations:** ^1^Department of Neurosurgery, Kaohsiung Chang Gung Memorial Hospital and Chang Gung University College of Medicine, Kaohsiung, Taiwan; ^2^Department of Trauma Surgery, Kaohsiung Chang Gung Memorial Hospital and Chang Gung University College of Medicine, Kaohsiung, Taiwan

## Abstract

**Introduction:**

Skull fractures are often found in patients with traumatic brain injury (TBI). Although skull fractures may indicate greater force impact and are associated with local or diffuse brain injuries, the prognostic value of skull fractures remains unclear. This retrospective study aimed to assess the association between skull fractures and mortality in patients with TBI.

**Methods:**

This study included 5,430 TBI patients registered in the trauma registry system from January 2009 to December 2018. Clinical and demographic data including age, sex, trauma mechanisms, comorbidities, Glasgow Coma Scale (GCS) score, abbreviated injury score (AIS)-head, injury severity score (ISS), and in-hospital mortality were acquired. Multiple logistic regression and propensity score matching were used to elucidate the effect of skull fractures on mortality outcomes of TBI patients.

**Results:**

Compared to TBI patients without skull fracture, patients with skull fractures were predominantly male, younger, had lower GCS upon arrival at the emergency room, and had higher AIS-head, ISS, and in-hospital mortality. The patients with skull fracture had 1.7-fold adjusted odds of mortality (95% confidence interval (CI): 1.27–2.25; *p* < 0.001) than those without skull fracture, controlling for age, sex, comorbidities, and AIS-head. Additionally, the propensity score-matched analysis of 1,023 selected paired patients revealed that skull fracture was significantly associated with increased 1.4-fold odds of risk for mortality (95% CI: 1.02–1.88; *p*=0.036).

**Conclusions:**

Using a propensity score-matched cohort to attenuate the confounding effect of age, comorbidities, and injury severity, skull fracture was identified as a significant independent risk factor for mortality in patients with TBI.

## 1. Introduction

Traumatic brain injury (TBI) is one of the leading causes of morbidity and mortality associated with road traffic accidents [1]. Currently, computed tomography (CT) has become the standard for initial evaluation of patients suspected with TBI, and skull fractures are often found in patients with TBI. It has been estimated that out of 4,660 patients with TBI, 28% of patients had skull fractures. In addition, skull fractures are found in 25% of patients with fatal head injuries at autopsy [2].

The article "The Association between Skull Bone Fractures and the Mortality Outcomes of Patients with Traumatic Brain Injury" was published in 2022. Journal: Emerg Med Int.

The clinical importance of skull fractures has been reported in the literature; however, the prognostic value of skull fractures remains unclear. Simulation data showed that skull fractures could reduce the risk of diffuse brain injury, but increase the risk of brain contusion [3]. Skull fractures have been reported to contribute to unfavorable outcomes in moderate [4] or severe TBI [5] and increase the risk of leakage of cerebrospinal fluid [6]. Additionally, skull fractures have been associated with local or diffuse injuries of the brain, including cranial nerve injury, seizures, and intracranial hemorrhage [2]. It has also been reported that associated neurologic deficits and complications are more common in patients with skull fractures than in patients without skull fractures [7].

Of note, the comorbidity and demographic features of patients, as well as trauma severity, may confound the assessment regarding the effect of skull fracture on mortality in patients with TBI. For example, aging is associated with a decrease in skull bone stiffness and may increase the occurrence of skull fractures [8]. Furthermore, women were suggested to have favorable outcomes with better recovery than men [9], and this effect is suggested to result from higher levels of circulating estrogen and progesterone [10–14]. In patients with liver cirrhosis, an increased risk of sustaining skull fracture was found to be 1.75 [15]. Meanwhile, the comorbidities of patients and an associated higher injury severity score (ISS) were also associated with increased mortality in patients with TBI [16].

To assess the effect of skull fracture on the mortality of patients with TBI, the present study was designed to investigate the relationship via a propensity score-matched cohort analysis of the registered data to attenuate the confounding effects of the associated comorbidities, demographic features, and injury severity of patients.

## 2. Methods

### 2.1. Ethics Statement

This study was approved by the Institutional Review Board (IRB) of Chang Gung Memorial Hospital (approval number 202000057B0). Because the study was designed for retrospective analysis of the registered database, the need for informed consent was waived according to IRB regulations.

### 2.2. Patient Population and Retrieved Information

We collected the medical data of 35,154 patients (Figure 1) between January 2009 and December 2018 from the trauma registry system of a level I trauma center in Southern Taiwan [17–20]. Only hospitalized adult patients (age ≥20 years) with TBI were included in this study. The abbreviated injury score (AIS) was used to evaluate injury severity in the following body regions: head/neck, face, chest, abdomen, extremities (including pelvis), and external region [21]. The AIS was a simplified, expert-based anatomical scale for the severity of bodily injuries, including traumatic brain injury [22, 23] with AIS = 1–6 points for injuries based on mortality probability. An injury with AIS = 1 is never fatal, while an injury AIS = 6 is almost certainly fatal. The ISS was calculated by summing the squares of the three highest AIS scores in each body region [24, 25] and was categorized into groups of 1–15 (mild to moderate), 16–24 (severe), and >24 (critical). Patients with multiple trauma (AIS ≥3 in other body regions besides the head) (*n* = 1,457), aged less than 20 (*n* = 683), burn injury (*n* = 2), or incomplete data (*n* = 0) were excluded. The retrieved patient information included age, sex, comorbidities cerebrovascular accident (CVA), hypertension (HTN), coronary artery disease (CAD), congestive heart failure (CHF), diabetes mellitus (DM), and end-stage renal disease (ESRD)), trauma mechanisms, Glasgow Coma Scale (GCS) score upon arrival at the emergency department, AIS, ISS, hospital length of stay (LOS), and in-hospital mortality. According to the GCS, the severity of TBI was categorized in terms of mild (13–15), moderate (9–12), and severe (<8) injuries [26].

The article "The Association between Skull Bone Fractures and the Mortality Outcomes of Patients with Traumatic Brain Injury" was published in 2022. Journal: Emerg Med Int.

### 2.3. Statistical Analysis

Patient characteristics are summarized as mean ± standard deviation, median with interquartile range (GCS and ISS), or frequency (%) as appropriate. Demographic traits and clinical variables were compared between the two groups of patients (those with skull fracture versus without skull fracture) using the chi-square test. In this study, the primary outcome measure was in-hospital mortality. The adjusted odds ratio of mortality was calculated using logistic regression, controlling for age, sex, comorbidities, and AIS-head. Independent risk factors for mortality were evaluated via univariate and multivariate logistic regressions, which included parameters that were significant in the univariate model. In addition, a selected cohort was studied with propensity score matching of parameters with significance in multivariate logistic regression to evaluate the effect of skull fracture on mortality. All analyses were performed using the SPSS software (IBM, version 23). A 1 : 1 propensity score-matched study population was created by the greedy method using the *R* software (version 3.5.0; package: MatchIt, method: match it) with a 0.2 caliper width to attenuate the influence of confounding variables on the outcome assessment. A *p* value of <0.05 was set to determine statistically significant group differences.

The article "The Association between Skull Bone Fractures and the Mortality Outcomes of Patients with Traumatic Brain Injury" was published in 2022. Journal: Emerg Med Int.

## 3. Results

As given in Table 1, a total of 5,430 patients who were sent to our emergency room, including 3,279 men (60.4%) and 2151 women (39.6%), were included in this study. The mean age at the time of the accident was 55.1 ± 19.6 years. The most commonly encountered trauma mechanisms were motorcycle accidents (*n* = 2,844, 52.4%), followed by fall accidents (*n* = 1,732, 31.9%). Of these patients, 1,058 (19.5%) had skull fractures according to radiographic reports. HTN and DM were the first and second most common comorbidities, respectively, of these patients. Most patients presented with mild TBI with a GCS score of 13–15 (75.9%) and sustained an ISS <25 (90.2%). Of the patients with TBI, the median head AIS score was 4, and the average in-hospital mortality rate was 6.5%.

With male sex predominance, the average age was significantly lower in the skull fracture group than in the nonskull fracture group (Table 1). Significant differences in comorbidities and trauma mechanisms were also observed between patients with and without skull fractures. The GCS upon arrival at the emergency room was significantly lower in the skull fracture group than in the nonskull fracture group (median (Q_1_–Q_3_): 14 (9–15) vs. 15 (13–15); *p* < 0.001). Patients with skull fracture were also associated with higher ISS (16 (13–20) vs. 14 (9–16); *p* < 0.001), AIS-head (4 (3-4) vs. 3 (2–4); *p* < 0.001), mortality (10.3% vs. 5.6%; *p* < 0.001), and hospital stay (12.3 days vs. 10.4 days, *p* < 0.001) than those without skull fractures. The patients with skull fracture had 1.7-fold adjusted odds of mortality (95% CI: 1.27–2.25; *p* < 0.001) than those without skull fracture, under conditions controlled by age, sex, comorbidities, and AIS-head.

Table 2 provides the regression analysis of the associated risk of mortality by the presence of skull fracture, sex, age, comorbidities, AIS of head = 4, AIS of head = 5, and ISS. In univariate analysis, skull fracture was significantly associated with mortality (odds ratio, 1.9; 95% CI: 1.52–2.44; *p* < 0.001). Age, CVA, HTN, CAD, and ESRD were also significantly associated with mortality in patients with TBI. AIS-head (OR (95% CI): 10.0 (8.06–12.35); *p* < 0.001) and ISS (1.3 (1.24–1.29); *p* < 0.001) were also the significant risk factors for mortality. These parameters affecting mortality were included in further multivariate analyses to clarify their independent effects on mortality in patients with TBI. Skull fracture had a significant effect on the increasing mortality rate (1.8 (1.35–2.48); *p* < 0.001). In addition, age (1.0 (1.01–1.02); *p*=0.002), CAD (2.1 (1.32–3.31); *p*=0.002), and ESRD (4.2 (2.46–7.04); *p* < 0.001), excluding CVA and HTN, were identified as the independent risk factors for mortality. No trauma mechanisms had been identified as the independent risk factors for mortality. AIS-head = 4 and 5 were also associated with a significantly higher mortality rate (AIS-head = 4, 4.5 (1.76–11.51); *p*=0.002 and AIS-head = 5, 88.4 (27.28–286.26); *p* < 0.001, respectively). In contrast, AIS-head = 3 and ISS were not found to be a significant risk factor for mortality in patients with TBI.

The article "The Association between Skull Bone Fractures and the Mortality Outcomes of Patients with Traumatic Brain Injury" was published in 2022. Journal: Emerg Med Int.

To clarify the importance of skull fractures on the mortality of patients with TBI, 1 : 1 propensity score-matched patient cohorts with the same number of patients (*n* = 1,023 for each group) were created (Table 3) to attenuate the influence of confounding variables on the outcome assessment. In the matched patient cohort, there were no significant differences in age, sex, comorbidities, and AIS-head of the patients. The propensity score-matched analysis revealed that skull fracture remained significantly associated with an increased risk of mortality (1.4 (1.02–1.88); *p*=0.036).

## 4. Discussion

This study revealed that various factors were associated with skull fracture, including sex, age, comorbidities, GCS, ISS, and AIS-head. Multivariate analysis revealed that skull fracture, age, CAD, ESRD, and AIS-head were the independent risk factors for mortality in patients with TBI. Notably, many factors contribute to the mortality of patients with TBI [27]. Therefore, a propensity score-matched cohort, attenuating the confounding effect of the above variables, was created for this study in the outcome assessment. We found that skull fracture was still significantly associated with a 1.4-fold increase in mortality risk in patients with TBI.

In this study, females accounted for a small proportion (25.9%) of skull fracture patients, which is consistent with the results of a previous study that revealed gender differences in head trauma [5, 28]. Our previous studies also reported that more males than females sustained TBI in road accidents [18, 29]. The study results did not identify gender as a significant risk factor for mortality, which is in accordance with reports from other studies [10–14]. However, the complex physiological and social factors, which may have contributed by the differences between males and females in terms of skull fractures, were not explored in the study. Hence, further work on this topic is encouraged.

Furthermore, the study results revealed that age was an independent factor for mortality in patients with TBI. This result is consistent with those of many reports demonstrating that age is an important risk factor for mortality at any given level of GCS and AIS-head [30, 31]. Notably, in this study, patients with skull fractures were younger than those without skull fractures. It has been reported that aging may lead to a decrease in the stiffness of cranial bones [8]; therefore, older individuals are more prone to fractures; however, since the impact force sustained in each patient during the accident was unknown, the association between age and occurrence of skull fracture would not be conclusive.

The article "The Association between Skull Bone Fractures and the Mortality Outcomes of Patients with Traumatic Brain Injury" was published in 2022. Journal: Emerg Med Int.

Comorbidities of patients with TBI are important factors that contribute to alterations in the clinical course and influence the short-term and long-term outcomes of patients [32–34]. This study found an association between CAD and ESRD and increased mortality in patients with TBI, a phenomenon that has been supported by many prior studies [6, 16, 35–37]. Furthermore, in this study, we found that AIS-head, but not ISS, is an independent factor for mortality in patients with TBI. ISS was significantly associated with mortality only in the univariate regression, but not in the multivariate regression. Although ISS reflects the severity of multiple traumas in an injured person, the input of AIS-head into the regression may, to a large extent, explain the mortality outcome [38] and lessen the influence of ISS on the mortality outcome. Similar reports have shown that multiple traumas have no role in the mortality of patients with severe head injury [39, 40] and the mortality of patients depends on the severity of the intracranial pathology, regardless of ISS [41].

This study has some limitations. First, the analysis was limited to data from a level I regional trauma center, and the conclusions may not be generalizable to other regions or countries. Second, the different skull fracture types such as linear/nondepressed/depressed/compound fractures may be associated with different trauma mechanisms [42] and prognosis [43]. However, the skull fracture types and their association with local hematoma or parenchymal injury were not recorded in the trauma registry system and thus may lead to bias in the outcome assessment. Third, this study was a retrospective study based on a trauma registry database, which could have led to selection bias. The parameters that could be selected from the registered database for outcome analysis were still limited, considering the complex interaction of various factors leading to mortality in patients with TBI. Fourth, some bias may exist considering that the CT characteristics of patients which may also affect the prognosis of traumatic brain injury were not studied as a parameter. Fifth, the use of the propensity score as the matching method to attenuate nonrandomized assignment of the study population on the outcome assessment rely on a correct model fit of the relationship between the propensity score and the outcome [44, 45]. The goodness-of-fit for the propensity score model may have impact on the outcome evaluation [44, 45]. Furthermore, only short-term in-hospital mortality was measured, and long-term mortality was not included; thus, a selection bias may exist in the outcome analysis.

The article "The Association between Skull Bone Fractures and the Mortality Outcomes of Patients with Traumatic Brain Injury" was published in 2022. Journal: Emerg Med Int.

## 5. Conclusions

Using a propensity score-matched cohort to attenuate the confounding effect of age, comorbidities, and injury severity, skull fracture was identified as a significant independent risk factor for mortality in patients with TBI.

## Figures and Tables

**Figure 1:** Flowchart illustrating the enrollment of the adult patients with traumatic brain injuries in this study.

**Table 1:** The demographic traits and clinical characteristics of patients with traumatic brain injury.

Variables	All, *n* = 5430	Skull fracture (+), *n* = 1058	Skull fracture (−), *n* = 4372	OR (95% CI)	*P*
Gender					<0.001
Male, *n* (%)	3279 (60.4)	784 (74.1)	2495 (57.1)		
Female, *n* (%)	2151 (39.6)	274 (25.9)	1877 (42.9)		
Age, mean (years)	55.1 ± 19.6	46.7 ± 19.0	57.1 ± 19.2		<0.001
Comorbidities, *n* (%)					
CVA	298 (5.5)	24 (2.3)	274 (6.3)		<0.001
HTN	1734 (31.9)	197 (18.6)	1537 (35.2)		<0.001
CAD	264 (4.9)	33 (3.1)	231 (5.3)		0.003
CHF	38 (0.7)	2 (0.2)	36 (0.8)		0.026
DM	911 (16.8)	98 (9.3)	813 (18.6)		<0.001
ESRD	135 (2.5)	12 (1.1)	123 (2.8)		0.002
Trauma mechanisms, *n* (%)					
Automobile	119 (2.2)	8 (0.8)	111 (2.5)		<0.001
Motorcycle	2844 (52.4)	643 (60.8)	2201 (50.3)		<0.001
Bicycle	275 (5.1)	50 (4.7)	225 (5.1)		0.576
Pedestrian	191 (3.5)	43 (4.1)	148 (3.4)		0.282
Fall	1732 (31.9)	249 (23.5)	1483 (33.9)		<0.001
Strike by against	269 (5.0)	65 (6.1)	204 (4.7)		0.047
GCS, median (IQR)	15 (13–15)	14 (9–15)	15 (13–15)		<0.001
3–8	788 (14.5)	259 (24.5)	529 (12.1)		<0.001
9–12	523 (9.6)	145 (13.7)	378 (8.6)		<0.001
13–15	4119 (75.9)	654 (61.8)	3465 (79.3)		<0.001
ISS, median (IQR)	16 (9–17)	16 (13–20)	14 (9–16)		<0.001
1–15	2551 (47.0)	328 (31.0)	2223 (50.8)		<0.001
16–24	2345 (43.2)	574 (54.3)	1771 (40.5)		<0.001
≥25	534 (9.8)	156 (14.7)	378 (8.6)		<0.001
AIS-head, median (IQR)	4 (3-4)	4 (3-4)	3 (2–4)		<0.001
Mortality	355 (6.5)	109 (10.3)	246 (5.6)	1.9 (1.52–2.44)	<0.001
Mortality (AOR)^*∗*^	—	—	—	1.7 (1.27–2.25)	<0.001
Hospital stay (days)	10.8 ± 11.7	12.3 ± 11.7	10.4 ± 11.7		<0.001

AIS, abbreviated injury score; AOR, adjusted odds ratio; CAD, coronary artery disease; CHF, congestive heart failure; CI, confidence interval; CVA, cerebral vascular accident; DM, diabetes mellitus; ESRD, end-stage renal disease; GCS, Glasgow Coma Scale; HTN, hypertension; IQR, interquartile range; ISS, injury severity score; OR, odds ratio. ^*∗*^AOR, controlled for age, sex, comorbidities, and AIS-head.

The article "The Association between Skull Bone Fractures and the Mortality Outcomes of Patients with Traumatic Brain Injury" was published in 2022. Journal: Emerg Med Int.

**Table 2:** Univariate and multivariate logistic regressions of the risk factors for mortality of the patients with traumatic brain injury.

Mortality	Univariate analysis			Multivariate analysis		
	OR	95% CI	*P*	OR	95% CI	*P*
Skull fracture (+)	1.9	1.52–2.44	<0.001	1.8	1.35–2.48	<0.001
Gender			0.157			
Male	1.2	0.94–1.47		—	—	
Female	0.9	0.68–1.06		—	—	
Age	1.0	1.02–1.03	<0.001	1.0	1.01–1.02	0.002
Comorbidities						
CVA	1.5	1.02–2.29	0.041	1.1	0.69–1.86	0.637
HTN	1.7	1.33–2.06	<0.001	1.1	0.81–1.49	0.541
CAD	2.8	1.93–3.92	<0.001	2.1	1.32–3.31	0.002
CHF	2.2	0.85–5.63	0.106	—	—	
DM	1.2	0.92–1.59	0.166	—	—	
ESRD	5.0	3.32–7.52	<0.001	4.2	2.46–7.04	<0.001
Trauma mechanisms						
Automobile	0.9	0.41–1.93	0.770	—	—	
Motorcycle	0.5	0.38–0.60	<0.001	0.8	0.51–1.34	0.442
Bicycle	1.7	1.12–2.51	0.013	1.5	0.80–2.91	0.203
Pedestrian	0.9	0.47–1.61	0.658	—	—	
Fall	2.1	1.66–2.57	<0.001	1.2	0.74–1.92	0.483
Strike by/against	0.7	0.41–1.26	0.248	—	—	
AIS-head						
AIS = 3	0.2	0.11–0.27	<0.001	2.2	0.89–5.46	0.087
AIS = 4	0.5	0.37–0.60	<0.001	4.5	1.76–11.51	0.002
AIS = 5	32.4	25.25–41.64	<0.001	88.4	27.28–286.26	<0.001
ISS	1.3	1.24–1.29	<0.001	1.0	0.97–1.06	0.568

CAD, coronary artery disease; CHF, congestive heart failure; CI, confidence interval; CVA, cerebral vascular accident; DM, diabetes mellitus; ESRD, end-stage renal disease; GCS, Glasgow Coma Scale; HTN, hypertension; ISS, injury severity score; OR, odds ratio.

**Table 3:** Propensity score-matched cohort of the patients with or without skull fracture.

Propensity score-matched cohort					
	Skull fracture (+), *n* = 1,023	Skull fracture (−), *n* = 1,023	OR (95% CI)	*P*	Standardized difference (%)
Age	47.0 ± 18.8	47.4 ± 18.7	—	0.646	−2.03
Male	757 (74.0)	757 (74.0)	1.0 (0.82–1.22)		0.00
Comorbidities					
CVA	21 (2.1)	21 (2.1)	1.0 (0.54–1.84)	1.000	0.00
HTN	192 (18.8)	192 (18.8)	1.0 (0.80–1.25)	1.000	0.00
CAD	29 (2.8)	29 (2.8)	1.0 (0.59–1.69)	1.000	0.00
CHF	1 (0.1)	1 (0.1)	1.0 (0.06–16.01)	1.000	0.00
DM	92 (9.0)	92 (9.0)	1.0 (0.74–1.35)	1.000	0.00
ESRD	5 (0.5)	5 (0.5)	1.0 (0.29–3.47)	1.000	0.00
AIS-head	3.6 ± 1.0	3.7 ± 1.0	—	0.678	−1.84
Mortality	105 (10.3)	78 (7.6)	1.4 (1.02–1.88)	0.036	—

AIS, abbreviated injury score; CAD, coronary artery disease; CHF, congestive heart failure; CI, confidence interval; CVA, cerebral vascular accident; DM, diabetes mellitus; ESRD, end-stage renal disease; HTN, hypertension; OR, odds ratio.

The article "The Association between Skull Bone Fractures and the Mortality Outcomes of Patients with Traumatic Brain Injury" was published in 2022. Journal: Emerg Med Int.

## Data Availability

No data were used to support this study.

## References

[1] Maas A. I. R., Menon D. K., Adelson P. D. (2017). Traumatic brain injury: integrated approaches to improve prevention, clinical care, and research. *The Lancet Neurology*.

[2] Hardman J. M., Manoukian A. (2002). Pathology of head trauma. *Neuroimaging Clinics of North America*.

[3] Ren L., Wang D., Liu X., Yu H., Jiang C., Hu Y. (2020). Influence of skull fracture on traumatic brain injury risk induced by blunt impact. *International Journal of Environmental Research and Public Health*.

[4] Fabbri A., Servadei F., Marchesini G., Stein S. C., Vandelli A. (2008). Early predictors of unfavourable outcome in subjects with moderate head injury in the emergency department. *Journal of Neurology, Neurosurgery & Psychiatry*.

[5] Tseng W. C., Shih H. M., Su Y. C., Chen H. W., Hsiao K. Y., Chen I. C. (2011). The association between skull bone fractures and outcomes in patients with severe traumatic brain injury. *The Journal of Trauma*.

[6] Liao C. C., Chiu W. T., Yeh C. C., Chang H. C., Chen T. L. (2012). Risk and outcomes for traumatic brain injury in patients with mental disorders. *Journal of Neurology, Neurosurgery & Psychiatry*.

[7] Wiederholt W. C., Melton L. J., Annegers J. F., Grabow J. D., Laws E. R., Ilstrup D. M. (1989). Short-term outcomes of skull fracture: a population-based study of survival and neurologic complications. *Neurology*.

[8] Torimitsu S., Nishida Y., Takano T. (2014). Statistical analysis of biomechanical properties of the adult skull and age-related structural changes by sex in a Japanese forensic sample. *Forensic Science International*.

[9] Wohltmann C. D., Franklin G. A., Boaz P. W. (2001). A multicenter evaluation of whether gender dimorphism affects survival after trauma. *The American Journal of Surgery*.

[10] Hu Z., Li Y., Fang M., Wai M. S., Yew D. T. (2009). Exogenous progesterone: a potential therapeutic candidate in CNS injury and neurodegeneration. *Current Medicinal Chemistry*.

[11] Roof R. L., Hall E. D. (2000). Gender differences in acute CNS trauma and stroke: neuroprotective effects of estrogen and progesterone. *Journal of Neurotrauma*.

[12] Sayeed I., Stein D. G. (2009). Progesterone as a neuroprotective factor in traumatic and ischemic brain injury. *Progress in Brain Research*.

[13] Stein D. G. (2001). Brain damage, sex hormones and recovery: a new role for progesterone and estrogen?. *Trends in Neurosciences*.

[14] Stein D. G., Sayeed I. (2010). Is progesterone worth consideration as a treatment for brain injury?. *American Journal of Roentgenology*.

The article "The Association between Skull Bone Fractures and the Mortality Outcomes of Patients with Traumatic Brain Injury" was published in 2022. Journal: Emerg Med Int.

[15] Ezaz G., Murphy S. L., Mellinger J., Tapper E. B. (2018). Increased morbidity and mortality associated with falls among patients with cirrhosis. *The American Journal of Medicine*.

[16] Shibahashi K., Sugiyama K., Okura Y., Hoda H., Hamabe Y. (2017). Multicenter retrospective cohort study of “talk and die” after traumatic brain injury. *World Neurosurgery*.

[17] Hsieh C. H., Chen Y. C., Hsu S. Y., Hsieh H. Y., Chien P. C. (2018). Defining polytrauma by abbreviated injury scale ≥3 for a least two body regions is insufficient in terms of short-term outcome: a cross-sectional study at a level I trauma center. *Biomedical Journal*.

[18] Hsieh C. H., Hsu S. Y., Hsieh H. Y., Chen Y. C. (2017). Differences between the sexes in motorcycle-related injuries and fatalities at a Taiwanese level I trauma center. *Biomedical Journal*.

[19] Hsieh C. H., Liu H. T., Hsu S. Y., Hsieh H. Y., Chen Y. C. (2017). Motorcycle-related hospitalizations of the elderly. *Biomedical Journal*.

[20] Su W. T., Wu S. C., Huang C. Y. (2020). Geriatric nutritional risk index as a screening tool to identify patients with malnutrition at a high risk of in-hospital mortality among elderly patients with femoral fractures-a retrospective study in a level I trauma center. *International Journal of Environmental Research and Public Health*.

[21] Hsu S. Y., Wu S. C., Rau C. S. (2019). Impact of adapting the abbreviated injury scale (AIS)-2005 from AIS-1998 on injury severity scores and clinical outcome. *International Journal of Environmental Research and Public Health*.

[22] Foreman B. P., Caesar R. R., Parks J. (2007). Usefulness of the abbreviated injury score and the injury severity score in comparison to the glasgow coma scale in predicting outcome after traumatic brain injury. *The Journal of Trauma, Injury, Infection, and Critical Care*.

[23] Rau C. S., Kuo P. J., Chien P. C., Huang C. Y., Hsieh H. Y., Hsieh C. H. (2018). Mortality prediction in patients with isolated moderate and severe traumatic brain injury using machine learning models. *PLoS One*.

[24] Baker S. P., O’Neill B. (1976). The injury severity score: an update. *The Journal of Trauma, Injury, Infection, and Critical Care*.

[25] Baker S. P., O’Neill B., Haddon W., Long W. B. (1974). The injury severity score: a method for describing patients with multiple injuries and evaluating emergency care. *The Journal of Trauma, Injury, Infection, and Critical Care*.

[26] Teasdale G., Jennett B. (1974). Assessment of coma and impaired consciousness. a practical scale. *The Lancet*.

[27] MRC CRASH Trial Collaborators, Arango M., Yutthakasemsunt S. (2008). Predicting outcome after traumatic brain injury: practical prognostic models based on large cohort of international patients. *BMJ*.

The article "The Association between Skull Bone Fractures and the Mortality Outcomes of Patients with Traumatic Brain Injury" was published in 2022. Journal: Emerg Med Int.

[28] Jaja B. R., Eghwrudjakpor P. O. (2014). Effect of demographic and injury etiologic factors on intensive care unit mortality after severe head injury in a low middle income country. *Annals of African Medicine*.

[29] Tang C. E., Liu H. T., Kuo P. J. (2018). Impact of sexual dimorphism on trauma patterns and clinical outcomes of patients with a high-risk score of the osteoporosis self-assessment tool for asians: a propensity score-matched analysis. *International Journal of Environmental Research and Public Health*.

[30] Demetriades D., Kuncir E., Murray J., Velmahos G. C., Rhee P., Chan L. (2004). Mortality prediction of head abbreviated injury score and glasgow coma scale: analysis of 7, 764 head injuries. *Journal of the American College of Surgeons*.

[31] Mosenthal A. C., Lavery R. F., Addis M. (2002). Isolated traumatic brain injury: age is an independent predictor of mortality and early outcome. *The Journal of Trauma, Injury, Infection, and Critical Care*.

[32] Feinstein A. R. (1970). The pre-therapeutic classification of CO-morbidity in chronic disease. *Journal of Chronic Diseases*.

[33] Soo M., Robertson L. M., Ali T. (2014). Approaches to ascertaining comorbidity information: validation of routine hospital episode data with clinician-based case note review. *BMC Research Notes*.

[34] Young J. S., Hobbs J. G., Bailes J. E. (2016). The impact of traumatic brain injury on the aging brain. *Current Psychiatry Reports*.

[35] Ahmadi N., Hajsadeghi F., Yehuda R. (2015). Traumatic brain injury, coronary atherosclerosis and cardiovascular mortality. *Brain Injury*.

[36] Dams-O’Connor K., Gibbons L. E., Landau A., Larson E. B., Crane P. K. (2016). Health problems precede traumatic brain injury in older adults. *Journal of the American Geriatrics Society*.

[37] Thompson H. J., Dikmen S., Temkin N. (2012). Prevalence of comorbidity and its association with traumatic brain injury and outcomes in older adults. *Research in Gerontological Nursing*.

[38] Davis D. P., Kene M., Vilke G. M. (2007). Head-injured patients who “talk and die”: the San Diego perspective. *The Journal of Trauma, Injury, Infection, and Critical Care*.

[39] Facco E., Zuccarello M., Pittoni G. (1986). Early outcome prediction in severe head injury: comparison between children and adults. *Child’s Nervous System: ChNS*.

[40] Levati A., Farina M. L., Vecchi G., Rossanda M., Marrubini M. B. (1982). Prognosis of severe head injuries. *Journal of Neurosurgery*.

[41] Baltas I., Gerogiannis N., Sakellariou P., Matamis D., Prassas A., Fylaktakis M. (1998). Outcome in severely head injured patients with and without multiple trauma. *Journal of Neurosurgical Sciences*.

The article "The Association between Skull Bone Fractures and the Mortality Outcomes of Patients with Traumatic Brain Injury" was published in 2022. Journal: Emerg Med Int.

[42] Saadat S., Rashidi-Ranjbar N., Rasouli M. R., Rahimi-Movaghar V. (2011). Pattern of skull fracture in Iran: report of Iran national trauma project. *Turkish Journal of Trauma and Emergency Surgery*.

[43] Yanagawa Y., Sakamoto T., Saitoh D. (2000). Significance of shock in head-injured patients with skull fracture. *Neurologia Medico-Chirurgica*.

[44] Austin P. C. (2008). Goodness-of-fit diagnostics for the propensity score model when estimating treatment effects using covariate adjustment with the propensity score. *Pharmacoepidemiology and Drug Safety*.

[45] Austin P. C. (2011). An introduction to propensity score methods for reducing the effects of confounding in observational studies. *Multivariate Behavioral Research*.

